# Drinking Water Sources along the Banks of Buriganga River of Bangladesh are Polluted and Possess Serious Health Risks: A Comprehensive In Vivo Analysis

**DOI:** 10.1155/2023/3369163

**Published:** 2023-01-11

**Authors:** Banna Ghosh, Muhammed Mahfuzur Rahman, Tanoy Saha, Md. Jamal Hossain, Safaet Alam, D. A. Anwar Al-Aman, Md. Shahidulla Kayser, Md. Shariful Islam, Md. Kamrul Islam, Amit Singh, Tufael Ahmed

**Affiliations:** ^1^Department of Pharmacy, State University of Bangladesh, 77 Satmasjid Road, Dhanmondi, Dhaka 1205, Bangladesh; ^2^Drugs and Toxins Research Division, BCSIR Laboratories Rajshahi, Bangladesh Council of Scientific and Industrial Research, Rajshahi 6206, Bangladesh

## Abstract

**Background:**

The river Buriganga, one of the major dumping zones of industrial wastes in Bangladesh, is responsible for contaminating the drinking water sources along its length. This study aimed to assess the water quality from these sources by monitoring the changes in hematological, biochemical, and histological parameters caused in healthy rats due to their consumption.

**Methods:**

Using ethylenediaminetetraacetic acid (EDTA) as an anticoagulant agent, hematological and biochemical analyses of Sprague–Dawley rat models were executed in this study. Following blood sampling, the rats were sacrificed, and the heart, lungs, kidneys, liver, and spleen were separated to carry out the histological analysis. Later, to perform the statistical analysis, SPSS, V.25.0 was utilized.

**Results:**

A significant rise (*p* < 0.02) in body weight was recorded due to increased protein synthesis, inflammations; increased lymphocyte, white blood cell (WBC), and neutrophil count but hemoglobin (20.0 ± 1.39 g/dL vs. 15.25 ± 0.36 g/dL; *p*) and red blood cell (RBC) count ((6.24 ± 0.45) × 10^6^/µL vs. (5.47 ± 0.34) × 10^6^/µL)) decreased due to infections and hematopoietic stem cell poisoning by pathogens in water samples. Elevated (*p* < 0.01) serum urea, creatinine, alanine, and aspartate aminotransferase levels indicated kidney malfunction and hepatic tissue necrosis. Histological analysis revealed gross lesions, internal hemorrhages in the brain; inflammations, granulomas, migrating macrophages in the spleen; fibrosis (resulting in hypo-perfusion), and collagen formation in cardiac muscles.

**Conclusions:**

The findings in this study provide comprehensive evidence, based on *in vivo* analysis, that the water bodies around the Buriganga river are likely to be contaminated with toxic chemicals and microbial entities making them unfit for human consumption.

## 1. Introduction

Dhaka city, the capital of Bangladesh, is surrounded by four rivers. Balu on the east; Tongi Khal on the north; Turag on the west; and Turag-Buriganga on the south [1]. All of them are extensively polluted and have been charged with containing toxic effluents, chemical wastes, elevated levels of heavy metals, fertilizers, pesticides, and so on [1, 2]. The Buriganga River, regarded as the most significant of all, is considered Dhaka's lifeline. This 18 km long river, situated in the south of the city, has become the water source used by the city residents for bathing, drinking, irrigation, and industrial purposes [1]. However, parallel to domestic wastes, 627 dyeing, 343 tanneries, and 104 fertilizer industries discharge untreated industrial effluents daily, covering 5000 to 9000 m^2^ of the river body [3, 4]. Because of a large number of pollutants discharged, the Buriganga River is getting worse. Furthermore, man-made activities such as cleaning, washing, bathing, and so on pollute the river's water. In recent years, many studies have shown widespread metallic water contamination with metals, including As, Fe, Mn, Cu, Cd, Cr, Pb, Ni, Zn, and others being found in the contaminated water in various concentrations [5]. Epoxy, polyurethane, enamel, ductile-silver white metal, hydrochloric acid, alkalis, lime, caustic soda, aluminum, zinc chromate, zinc phosphate, asbestos, and other toxic materials have all been identified in the effluents of the river water [4]. Chlorides, pH, dissolved oxygen, biological oxygen demand, and other water quality indicators seldom meet the requirements established by the Bangladeshi Department of Environment [6].

The Buriganga river was long ago designated as a “waste dump” that could not sustain aquatic life and whose water is exceptionally unsafe for home use. In addition, drinking water pipes are frequently leaking into the sewer systems in Dhaka, exposing millions of people to the river's contaminated water and seriously endangering their health [3]. Metals are regarded as poisons and eventually affect the body when consumed in higher than recommended amounts. Several metals such as lead, cadmium, chromium, and arsenic may not have any substantial benefits for the body, but they do directly harm the liver and kidney, and even at normal levels, they are highly nephrotoxic and hepatotoxic [7]. Besides, Lead intoxication can cause damage to the brain and nerves. It also slows enzymes and is harmful to many different metabolic processes [8]. Like this, manganese toxicity can cause manganism, a chronic neurological condition characterized by tremors, trouble walking, and facial muscle spasms. These symptoms are frequently followed by less severe ones such as aggression, impatience, and hallucinations. There is no doubt that industrial pollution and water contamination are related [9]. According to a recent health benefits assessment, industrial exposures may be responsible for up to 10% of end-stage renal disease and various liver illnesses [10]. Specifically, according to a recent study, the Buringa water had high levels of phosphate (PO4^−3^), ammonia, organic matter, biological oxygen demand (BOD), and chemical oxygen demand (COD). The study also highlighted the serious risks to public health and the potential harm to the environment [6].

Due to several risk factors, research has long been interested in the Buriganga River's water quality and the water from nearby sources. Numerous studies have been conducted in these areas to estimate the physicochemical parameters, presence of toxic wastes, heavy metals in drinking water, and possible sources of contamination [1, 4, 9, 11, 12]. However, little effort has been put forth to examine the risk of long-term use of such polluted water using animal models.

Hence, in this present study, water samples from the major drinking outlets around the Buriganga river were collected and fed to Sprague–Dawley rats in the laboratory over 56 days. The animals were later sacrificed; blood and tissue samples were collected to investigate changes in biochemical, hematological, and histological parameters. These assessments could provide evidence that would clarify the impact of (if any) Buriganga river water on the health-related issues of the population living along the length of the river. Thus, the objectives of this study were to examine the hematological, biochemical parameters, and tissue histology of some major organs of Sprague–Dawley rats fed with the contaminated water and estimate the significance of the change in physiology made due to long-term exposure to the sampled drinking water.

## 2. Materials and Methods

Test water samples were randomly collected from different sites (Sadarghat, Tanti Bazar, Shakhari Bazar, Islampur, Nowab bari Ghat, and Badamtoli Bridge) covering the length of Buriganga, following the method of Sunjida, et al. 2016 [9]. At each point, a total of 10 samples were taken from chlorine-treated groundwater sources (tap water) and collected in double-capped polyethylene bottles previously washed with detergent, dilute HNO_3,_ and Milli *Q* Water (MQW). A total of 12 healthy, eight weeks old, female albino, Sprague–Dawley rats, weighing 160 ± 25 g, were housed in plastic (30 × 20 × 13 cm) cages; kept at laboratories where room temperature and relative humidity (25°C, 60%) were strictly monitored. All experimentations associated with living subjects were performed according to the institutional guidelines for animal experimentation of the Department of Pharmacy, State University of Bangladesh. Besides, the Animal Ethics committee of the State University of Bangladesh has critically reviewed and approved the study protocols and detailed guidelines. The Federation of European Laboratory Animal Science Associations (FELASA) guidelines and recommendations were followed to reduce the pain and stress of the experimental animal. The subjects were kept for one week in order to settle into their new environment. Later, they were divided into two groups of 6 members, and all were fed and allowed to drink water ad libitum. Group 2 (the experimental group) received the sample water, while Group 1 served as the control group and was given normal drinking water. All the individual rats in both groups were marked (as I, II, III, IV, V, and VI) carefully on the tail for ease of identification and these identification marks were used to record the responses of an individual rat prior to and during the experiment. The experimental study was conducted for 56 consecutive days. The body weight of each rat in the treatment and control group was measured at the beginning of the experiment using an electronic analytical weight balance. Two times measurements of weight per week were recorded during the total exposure period. After 56 days of exposure, the rats were fasted overnight and weighed. Blood samples were collected from every individual rat through cardiac puncture using a 5 mL syringe with a 25 G needle and immediately transferred to a tube containing 8.5% of the anticoagulant ethylenediaminetetraacetic acid (EDTA) [13]. Samples were immediately transferred to anticoagulant-containing tubes and mixed with 8.5% EDTA. All the tubes were properly labeled and immediately transferred to the laboratory for hematological and biochemical analysis.

At the end of the experiment, an anesthesia overdose (Ketamine HCl (100 mg/kg) and xylazine (7.5 mg/kg) through the intraperitoneal route were given to the rat models followed by euthanasia [14]. The heart, lungs, kidneys, liver, and spleen from each rat were removed using a sharp blade and scissors, immediately rinsed with physiological saline, blotted, dried, and later weighed. The organs were separately preserved in 10% formaldehyde (pH 7.2 to 7.4), and sections of tissues were sliced later for histological analysis [15].

All the hematological and biochemical analyses were performed using the laboratory facility at the Pharmacology research laboratory, Jahangirnagar University, Savar, Dhaka. The hematological analyzed parameters were white blood cell (WBC) count, red blood cell (RBC) count, hemoglobin concentration (Hb), mean corpuscular hemoglobin (MCH), mean corpuscular volume (MCV), mean corpuscular hemoglobin concentration (MCHC), and platelet count (PLT). The biochemical parameters were serum urea, creatinine, bilirubin, aspartate aminotransferase (AST), and alanine aminotransferase (ALT) levels [16, 17].

For the histological evaluations, the organs were trimmed to 0.5 cm in thickness and placed in cassettes. The cassettes were submerged in 10% formalin solution overnight, before undergoing a series of dehydration processes for about 16 hr in an automated processor (Leica ASP300, Germany). The samples were then embedded with paraffin to form a block by a processor machine (Leica EG1160, Germany) and left to cool. The blocks were trimmed to about 3–5 *μ*m in thickness using a sectioning rotary microtome (Leica RM2155, Germany) and directly placed in a 45°C water bath before mounting on slides. All the glass slides were labeled with a diamond pen and mounted on a hot plate (54°C) overnight. Finally, after staining with hematoxylin and eosin (H&E) the samples were examined under a light microscope at different magnifications, and images (1360 × 1024 pixels each image) were captured using 100 times magnification [18].

Statistical analysis was performed on a PC using SPSS, V.25.0. All the parameters were recorded in triplicates and expressed as mean ± SEM of *n* experiments (where *n* represents the number of animals used). Values between the control and the experimental group were compared using the *t*-test and *p* values lower than 0.05 were considered to be statistically significant.

## 3. Results

After 56 days, significant (*p* < 0.001) variations in body weight were found between the sample and control group. The mean body weight of the rats in the test group (137 ± 1.0 mg) was higher compared to the rats in the control group (121.8 ± 1.2 mg) (Figure 1).

Hematological analysis revealed a significant difference only in the hemoglobin level (*p* < 0.01) of the test animals which was 4.75 ± 1.75 mg higher than the control group. Other parameters such as the values of MCV, MCH, MCHC, and PCV were comparable in both groups. There was a reduction in the RBC and platelet count while the lymphocytes such as WBC, monocyte, eosinophil, basophil, and neutrophil counts increased (Table 1). In the biochemical analysis, significant variations were recorded in all the parameters being measured between the two groups of animals. Serum urea (*p* < 0.01) levels were 6.9 ± 2.04 mg/dL elevated and creatinine (*p* < 0.05) levels increased by 0.24 ± 0.09 mg/dL in the sample group animals. Both the concentrations of AST (*p* < 0.01) and ALT (*p* < 0.05) were found to be higher by 39.3 ± 13.8 and 5.92 ± 2.54 mg/dL, respectively, after the rats were in exposure to the sampled water (Figure 2).

All the values are expressed as mean ± SEM (*n* = 6). *p* < 0.05 significant when compared to the control group (normal water). Here, ^*∗*^*p* < 0.05, ^*∗∗*^*p* < 0.01 and ^*∗∗∗*^*p* < 0.001 when compared with the control group. Here, ESR = erythrocyte sedimentation rate; PCV = packed cell volume; MCV = mean corpuscular volume; MCH = mean corpuscular hemoglobin; MCHC = mean corpuscular hemoglobin concentration; RDW = red blood cell distribution width; WBC = white blood cell; RBC = red blood cell.

Histological analysis of the brain tissue revealed the presence of a gross lesion and mild-to-moderate focal hemorrhage in the sample group while the control group had normal brain histology (Figures 3(a) and 3(b)). Cardiac tissue from the rats receiving the sample water showed highly distorted cardiac muscle fibers with an increased collagen bundle (Figures 3(g) and 3(h)). Histological sections of the liver had sinusoidal dilatation, cytoplasmic vacuolation, and inflammation (Figures 3(c) and 3(d)). Renal tissue samples from the experimental groups had tissue degeneration at the glomerular tuft accompanied by lymphocyte infiltration. Additionally, the renal tubules were vacuolated and had lost their brush borders. The cells of both renal corpuscle and renal tubules lost a considerable amount of total protein as well. However renal tissue samples from the control group exhibited no such changes (Figures 3(i) and 3(j)). No visible changes were seen in the lung tissue sample from the two groups (Figures 3(e) and 3(f)) but a histological study of the spleen tissue revealed the presence of granulomas in the capsule and red pulp composed predominantly of infiltration of macrophages and rare lymphocytes and plasmacytes (Figures 3(k) and 3(l)).

## 4. Discussion

Globally, the supply of fresh water is being lowered continuously due to resource overuse, population growth, and rapid industrialization [19]. Industrialized countries have good monitoring and remediation initiatives to counteract these issues, and health hazards in developing countries are on the rise, due to fewer initiative programs and poor management by the authorities [20]. Nevertheless, there has been a recent upsurge in concern among the general population making river pollution one of the main topics in the environmental issue of urban Dhaka [9]. As a result, numerous investigations have been conducted to assess the quality of major water bodies around the country, especially in industrialized areas. All of these studies provide strong evidence that the water in the rivers around Dhaka, i.e., Buriganga, is highly contaminated containing toxic industrial wastes, heavy metals, etc., threatening the health of local communities [9]. Our present study has taken a newer approach of expanding the field of investigation by studying the long-term toxic effect of drinking water contaminated by the Buriganga river water, in an animal model. Our findings regarding the hematological, biochemical parameters, and histological observations corroborate previous in vitro studies conducted on the water from Buriganga and other surrounding sources and provide comprehensive evidence that the drinking water sources nearby Buriganga are highly polluted and unfit for human consumption.

Enhancement of body weight in test animals after treatment with polluted drinking water has been recorded in the previous report [9], but no plausible explanation was provided. However, drinking water contaminated with heavy metals and carcinogens such as arsenic, cadmium, lead, benzene, and trichloroethylene has been associated with the increased weight of organs such as the liver, spleen, pancreas, and heart in several studies [21]. Similarly, chronic infections (caused by pathogens present in the contaminated water in this case) have also been linked to inflamed liver and spleen along with increased protein synthesis by these organs [22]. This elevated number of tissue inflammation and protein synthesis of various organs as a measure to counteract the pathogenic infestations caused by consuming polluted water could add up to the increase in total body weight. Hematological changes similar to this study have been published in other studies where test animals were treated with polluted water or by water contaminated with industrial wastes containing toxic heavy metals [23, 24]. The intake of the polluted water could have had intoxicated the internal organs which were also evident in the histological tissue analysis. This might cause inhibition of erythropoiesis in the hemopoietic organs, decreasing the RBC, PCV, and Hb count resulting in an anemic condition in the rats [25]. Hypoxic conditions could also result in the release of immature RBCs in the blood as a compensatory measure resulting in a decrease in MCV, MCH, and MCHC values [26]. The WBCs are the body's first line of defense against pathogens [27]. Elevated levels of these cells in the body indicate internal infections [28]. This infection could be initiated by pathogens entering the rats from the polluted drinking water. An increase in serum urea and creatinine level indicates an increase in the tubular reabsorption of urea and decreased creatinine clearance both caused by a reduction of renal blood flow also known as hypo-perfusion [29]. This reduction in blood flow could be the sign of any condition that leads to a decrease in effective circulating blood volume caused by any cardiac impairment (failure/injury) [30]. This cardiac injury was clearly evident in the histological analysis (Figure 3: H, red arrow). On the other hand, the increase in ALT (*p* < 0.05) and AST levels is directly related to progressive liver damage (Figure 3: C), tissue necrosis, or extensive breakdown of body tissue leading to the liberation of these enzymes into the blood [31]. The hemorrhage and the edema indicate a severe form of brain injury and tissue damage (indicated by an arrow in Figure 3: A). Furthermore, the hemorrhage could worsen the inflammation further contributing to brain injury [32–34]. This brain damage could be a result of increased oxidative stress in brain tissue. Oxidative stress could damage the membrane phospholipids and DNA nucleotides directly and also indirectly through the mediation of various cellular cascades [35–37]. Additionally, the large consumption of oxygen by brain tissues makes them more vulnerable to oxidative stress [36]. These reactive oxygen species (ROS) could enter the body through polluted water. In the brain, increased ROS causes oxidative damage to all cellular components. The muscle fibers appeared deformed due to adverse accumulation of collagen increasing tissue stiffness and causing cardiac fibrosis. This is characterized by decreased contractility and thereby impairing the overall performance of the heart [38]. Several mediators could be responsible for the induction of this collagen formation such as transforming growth factor-*β*1 (TGF-*β*1) and angiotensin-converting enzyme 2 (ACE2). [39, 40]. However, the relationship between cardiac fibrosis and contaminated water consumption could trigger those mediators, and still, further relationship needs to be established. All three of these observations have been linked with bacterial infection and provide evidence that the water samples were the primary source of pathogenic bacteria. For example, bacterial invasion results in inflammation due to immune response. In addition, sinusoidal inflammation is associated with inflammatory diseases [41]. Finally, cytoplasmic vacuolation is a very common morphological change undergone by cells after exposure to infectious pathogens [42]. The progressive damage of liver tissue is also supported by the elevated levels of ALT and AST in the blood serum mentioned previously. Chromium, arsenic, etc., very common in polluted water, have been found highly nephrotoxic and hepatotoxic even at normal levels [43]. The liver and kidney damage in the rats could be associated with these two heavy metals present in the drinking water samples. The formation of granulomas and migration of macrophages is a common response shown by the body when it tries to eliminate microbes or foreign matters [44]. These pathogens or foreign matters could easily invade healthy rats due to the consumption of contaminated water.

## 5. Conclusion

Interpretations of the physiological changes recorded in the current study suggest that the inhabitants living near Buriganga are at serious health risks such as respiratory infections, liver cirrhosis, renal impairment, various tissue necrosis, and toxicities. Long-term consumption could also give rise to health issues such as reduced immunity, anemia, and cardiac fibrosis as well as numerous tissue inflammations in humans. Even though some parameters, i.e., MCH, MCHC, and WBC count showed gradual changes for which general explanations have been proposed but these variations were not significant to draw any blatant conclusion. Therefore, this study also demands future in vivo studies with broadened sample area, size, and increased duration, in order to elucidate these changes, understand the mechanism of actions triggering them and clarify the public health associated risks due to exposure to this contaminated water. Furthermore, since the river is polluted from various sources, including domestic, industrial, and dyeing wastewater, it is essential to investigate the concentrations of primary pollutants, such as the kind and amount of dye, trace element types and amounts, and chemical and biological contaminants.

## Figures and Tables

**Figure 1:** Effect of tap water (sample water) (*n* = 6) on body weight of Sprague–Dawley Rats compared to control groups (normal water) (*n* = 6). The weights of the rats were measured every four days for 56 days, and weight change was calculated relative to the initial weight at day 0.

**Figure 2:** Biochemical changes of Sprague–Dawley rats after 56 days of exposure to different types of water (normal water (control) vs. tap (sample) water). (a) Changes in serum urea level; (b) Changes in serum creatinine level; (c) changes in serum ALT level; (d) changes in serum AST level; (e) changes in serum bilirubin level;^*∗∗*^compared with the control group, *p* < 0.005;^*∗*^compared with a control group, *p* < 0.05. Results are shown as mean ± SEM of *n* = 6 rats per group.

**Figure 3:** Representative photomicrographs of distal organs of rats after 56-day exposure to sample tap water. Photomicrographs of slices from the brain (a–b), liver (c–d), lung (e–f), heart (g–h), kidney (i–j), and spleen (k–l) stained with hematoxylin and eosin. (a) Normal brain architecture with well delineated cortical layers and neuronal cells; (b) in the experimental group (tap water), gross lesion (black arrow) and mild-to-moderate focal hemorrhage (red arrow) was observed; (c) normal liver architecture with normal hepatocytes and red cell stasis within the central vein and sinusoids; (d) experimental rat liver section showing sinusoidal dilatation, cytoplasmic vacuolation and inflammation; (e) sections of lungs of control rat; (f) sections lungs of experimental rats showed no differences; (g) well developed and normal distribution of cardiac muscle fibers; normal appearance of cardiac tissue of control rat; (h) highly distorted cardiac muscle fibers with increased collagen bundle (red arrow) observed in experimental group and the muscle fibers appears deformed due to adverse accumulation of collagen increasing tissue stiffness causing cardiac fibrosis; (i) normal histological features of kidney including glomerulus and tubules of control rat-glomeruli are normal and tightly filing the Bowman's capsule and renal tubules are lined with typical thick cubic epithelium; (j) kidney section of experimental groups had degeneration of the glomerular tuft with infiltration of lymphocytes and the renal tubules became vacuolated along with losing their brush borders; (k) normal histology of spleen, region of the periarterial lymphoid sheath of control rat; (l) spleen tissue sample of experimental rat revealed the presence of granulomas in the capsule and red pulp.

**Table 1:** Hematological values (mean ± SEM) of Sprague–Dawley rats (*n* = 6) after 56 days of the experiment.

Sl. No.	Parameters	Group 1 (control)	Group 2 (sample water)
1	Hemoglobin	20.0 ± 1.39 g/dL	15.25 ± 0.36^*∗∗*^ g/dL
2	ESR	4.5 ± 1.1 mm/hr	4.5 ± 0.76 mm/hr
3	PCV	33.21 ± 1.13%	33.08 ± 2.13%
4	MCV	53.56 ± 0.69 fL/red cell	53.48 ± 0.70 fL/red cell
5	MCH	19.13 ± 0.38 pg/cell	18.38 ± 0.21 pg/cell
6	MCHC	33.83 ± 0.80 g/dL	33.8 ± 1.27 g/dL
7	RDW-SD	30.63 ± 1.56%	32.4 ± 1.44%
8	MPV	6.62 ± 0.080 fL	7.21 ± 0.27 fL
9	RDW-CV	16.67 ± 0.54%	16.22 ± 0.66%
10	WBC	4500 ± 295.52/µL	5350 ± 689.32/µl
11	RBC	(6.24 ± 0.45) × 10^6^/µL	(5.47 ± 0.34) × 10^6^/µL
12	Lymphocyte	77.83 ± 2.71/µL	81.83 ± 1.60/µL
13	Monocyte	1.50 ± 0.22/µL	2.0 ± 0.45/µL
14	Eosinophil	0.02 ± 0.0025l/µL	0.02 ± 0.0041l/µL
15	Basophil	2.83 ± 0.60/µL	3.03 ± 0.45/µL
16	Neutrophil	15.5 ± 2.96/µL	17 ± 1.03/µL
17	Platelet	539200 ± 8063.91/µL	528400 ± 20523/µL

## Data Availability

Further raw data will be found from the corresponding authors upon reasonable request.
